# Cavernous Sinus Thrombosis and Blindness Complicating Dental Infection

**DOI:** 10.7759/cureus.21318

**Published:** 2022-01-17

**Authors:** Emily Ming Choo Ng, Othmaliza Othman, Li Yen Chan, Nor Akmal Bahari

**Affiliations:** 1 Ophthalmology, Universiti Kebangsaan Malaysia, Kuala Lumpur, MYS; 2 Ophthalmology, University Kebangsaan Malaysia, Kuala Lumpur, MYS; 3 Ophthalmology, Kuala Lumpur General Hospital, Kuala Lumpur, MYS

**Keywords:** proptosis, ophthalmoplegia, blindness, odontogenic infection, anticoagulation, cavernous sinus thrombosis

## Abstract

A 32-year-old gentleman with underlying hypertension presented with left eye ptosis and diplopia for two weeks. He also complained of the left eye progressive blurring of vision. One week of left-sided toothache, headache, and fever preceded these symptoms. He visited a dental clinic for the toothache and was prescribed oral metronidazole before scheduling tooth extraction. However, the disease progressed with ocular symptoms. On examination, his visual acuity was 20/20 on the right and perception to light on the left. The left eye pupil was sluggish, and relative afferent pupillary reflex was positive. There was partial ptosis, mild proptosis, and ophthalmoplegia involving cranial nerve III, IV, and VI over the left. Hypoesthesia over the left V1 region was also present. Bilateral anterior and posterior segments were unremarkable. Blood investigations revealed an elevated total white cell count and C- reactive protein. Hence, an urgent computed tomography of the brain was requested and demonstrated left cavernous sinus thrombosis with diffuse thickening and enhancement extended anteriorly to the left orbital apex. He was admitted for intravenous ceftriaxone and subcutaneous enoxaparin. He was hemodynamically stable and allowed home with new direct anti-coagulants. He sustained the permanent sequelae of a left blind eye and residual cranial nerve palsies despite the treatment.

## Introduction

Cavernous sinus thrombosis (CST) is a life-threatening condition secondary to severe head injuries, infection, or any health conditions that can cause venous stasis [1-2]. CST secondary to odontogenic origin has been reported in patients with active dental infection or following dental procedures [3-5]. The mortality rate has significantly reduced in the era of antibiotics and anticoagulation. However, the morbidity of the disease remains. Therefore, early recognition of the disease and prompt treatment are essential to reduce the likelihood of complications. We report a case of dental infection complicated with CST and unilateral blindness.

## Case presentation

A 32-year-old gentleman with underlying hypertension presented to the ophthalmology clinic with two weeks' onset of drooping of the left upper eyelid and double vision followed by a progressive blurring of vision of the left eye. He denied any history of head injury or sinus congestion. His symptoms preceded a week of left-sided toothache, headache, and fever. He visited a dental clinic and was prescribed a course of oral metronidazole 500mg four times daily for a week before scheduling for left lower third molar extraction. However, the disease progressed with ocular symptoms. He only sought further advice when there was a progressive blurring of vision.

On examination, he was alert and well-oriented. His visual acuity was 20/20 on the right eye and perception to light on the left eye. Left eye pupil was mid dilated and sluggish. The relative afferent pupillary reflex was markedly positive on the left eye. Left-sided partial ptosis, mild proptosis (Figure 1), and ophthalmoplegia (Figure 2) were present. There was also hypoesthesia in the division of V1. However, there was an absence of eyelids swelling, pulsation, or bruit. The intraocular pressure was 16mmHg for bilateral eyes, and bilateral optic discs and retinal vessels were normal. He was afebrile and systemic examinations were unremarkable.

**Figure 1:** Left eye with partial ptosis and proptosis.

**Figure 2:** Left eye with restricted eye movement at all gazes.

Blood investigations revealed an elevated white cell count of 11.5 x 109/L (6.0- 10.0) and C- reactive protein of 28.3 mg/L (5.0). An urgent computed tomography (CT) scan showed left CST with diffuse thickening and enhancement extended anteriorly to the left orbital apex (Figure 3). He was started on intravenous ceftriaxone 2g twice daily. He was referred to the Neuro-medical team for anticoagulation and co-management. Subcutaneous enoxaparin 60mg twice daily was commenced and has later switched to oral dabigatran 150mg twice daily upon discharge. The infected left lower third molar was extracted during the admission. Nasal endoscopic examination was unremarkable. He was hemodynamically stable and completed intravenous ceftriaxone for six days. He was allowed home with oral cefuroxime 250mg twice daily for a day and oral dabigatran 150mg twice daily for six months. There was no recurrence of CST post-treatment.

**Figure 3:** An axial CT scan view showing left cavernous sinus diffuse thickening with filling defect and enhancement extending anteriorly to the left orbital apex.

## Discussion

The cavernous sinus is an important bilateral interconnected sinus in the middle cranial fossa that drains the head and neck. It is closely related to cranial nerve III, IV, V1, and V2 at the lateral wall and cranial nerve VI, sympathetic fibers, and internal carotid artery within the sinus. As the cerebral venous system is valveless, infection from the head and neck such as sinusitis, otitis media, dental abscess, orbital cellulitis can quickly spread to the cerebral venous sinuses [6-8].

The ocular manifestations of CST may mimic orbital cellulitis, superior ophthalmic vein thrombosis, orbital apex syndrome, carotid-cavernous fistula, and superior orbital fissure syndrome. Therefore, clinicians should have a high index of suspicion of CST in patients with multiple ophthalmoplegia, proptosis, ptosis, fever, and sensory disturbance of ophthalmic and maxillary divisions [9-10]. The definite diagnosis has to be confirmed with CT or magnetic resonance imaging (MRI) of the brain. Our patient had a cavernous sinus thickening and filling defect suggestive of thrombus.

Although the disease mortality is lowered in the era of antibiotics, close monitoring is also crucial to prevent the infection from spreading to the contralateral cavernous sinus and brain. The use of anticoagulation is the mainstay in the treatment of CST as it can halt the thrombus propagation and minimize complications [11-13]. The patient sustained the permanent sequelae of a left blind eye and residual cranial nerve palsies due to his late presentation. Early recognition of the symptoms and immediate treatment has successfully halted the disease progression and minimized systemic complications. 

Vision loss in CST can be secondary to central retinal artery occlusion, ophthalmic vein occlusion, emboli or thrombosis of the carotid artery, ischemic optic neuropathy, toxic neuritis, or exposure to keratitis [14]. We postulate that our patient had posterior ischemic optic neuropathy as the optic disc was normal and the vessels were not tortuous or dilated.

Our patient was treated with broad-spectrum empirical intravenous antibiotics and subcutaneous enoxaparin, followed by oral dabigatran 150mg twice daily for six months. The ptosis and ophthalmoplegia improved, with the proptosis resolved with treatment. The use of new direct oral anti-coagulants (NOAC) such as rivaroxaban and dabigatran has gained popularity in venous thrombotic events. The efficacy and safety of NOAC versus conventional warfarin are comparable [15-16]. This article highlights the ocular manifestations of CST and its management.

## Conclusions

Cavernous sinus thrombosis is a rare yet potentially lethal condition. Though disease mortality reduces with antibiotics and anticoagulation, many patients recover with residual neuropathy, blindness, or keratitis. The clinical suspicion and early imaging on presentation led us to accurate diagnosis and early intervention. However, the guarded prognosis of the CST, in this case, may primarily be due to late presentation. Awareness of these potential sequelae of dental infection needs to be highlighted. 

## References

[1] Coutinho JM (2015). Cerebral venous thrombosis. J Thromb Haemost.

[2] Stam J (2003). Cerebral venous and sinus thrombosis: incidence and causes. Adv Neurol.

[3] Yun MW, Hwang CF, Lui CC (1991). Cavernous sinus thrombosis following odontogenic and cervicofacial infection. Eur Arch Otorhinolaryngol.

[4] Verma R, Junewar V, Singh RK, Ram H, Pal US (2013). Bilateral cavernous sinus thrombosis and facial palsy as complications of dental abscess. Natl J Maxillofac Surg.

[5] Okamoto H, Ogata A, Kosugi M, Takashima H, Sakata S, Matsushima T (2012). Cavernous sinus thrombophlebitis related to dental infection--two case reports. Neurol Med Chir (Tokyo).

[6] Cannon ML, Antonio BL, McCloskey JJ, Hines MH, Tobin JR, Shetty AK (2004). Cavernous sinus thrombosis complicating sinusitis. Pediatr Crit Care Med.

[7] Zanoletti E, Cazzador D, Faccioli C, Sari M, Bovo R, Martini A (2015). Intracranial venous sinus thrombosis as a complication of otitis media in children: critical review of diagnosis and management. Int J Pediatr Otorhinolaryngol.

[8] Ann J K, Sreedhar A, Jacob MC (2016). A case of cavernous sinus thrombosis complicating orbital cellulitis. Kerala J Ophthalmol.

[9] Ebright JR, Pace MT, Niazi AF (2001). Septic thrombosis of the cavernous sinuses. Arch Intern Med.

[10] Visvanathan V, Uppal S, Prowse S (2010). Ocular manifestations of cavernous sinus thrombosis. BMJ Case Rep.

[11] Saposnik G, Barinagarrementeria F, Brown RD Jr (2011). Diagnosis and management of cerebral venous thrombosis: a statement for healthcare professionals from the American Heart Association/American Stroke Association. Stroke.

[12] Coutinho J, de Bruijn SF, Deveber G, Stam J (2011). Anticoagulation for cerebral venous sinus thrombosis. Cochrane Database Syst Rev.

[13] Misra UK, Kalita J, Chandra S, Kumar B, Bansal V (2012). Low molecular weight heparin versus unfractionated heparin in cerebral venous sinus thrombosis: a randomized controlled trial. Eur J Neurol.

[14] Yassur I, Hirschbein MJ, Karesh JW (328-346). Ophthalmic considerations in oral and maxillofacial infections. Textbook of oral and maxillofacial infections, 4th edn.

[15] Ferro JM, Coutinho JM, Dentali F (2019). Safety and efficacy of Dabigatran Etexilate vs dose-adjusted warfarin in patients with cerebral venous thrombosis: a randomized clinical trial. JAMA Neurol.

[16] Wasay M, Khan M, Rajput HM (2019). New oral anticoagulants versus warfarin for cerebral venous thrombosis: a multi-center, observational study. J Stroke.

